# Effective molecular targeting of CDK4/6 and IGF-1R in a rare *FUS-ERG* fusion *CDKN2A*-deletion doxorubicin-resistant Ewing's sarcoma patient-derived orthotopic xenograft (PDOX) nude-mouse model

**DOI:** 10.18632/oncotarget.9879

**Published:** 2016-06-07

**Authors:** Takashi Murakami, Arun S. Singh, Tasuku Kiyuna, Sarah M. Dry, Yunfeng Li, Aaron W. James, Kentaro Igarashi, Kei Kawaguchi, Jonathan C. DeLong, Yong Zhang, Yukihiko Hiroshima, Tara Russell, Mark A. Eckardt, Jane Yanagawa, Noah Federman, Ryusei Matsuyama, Takashi Chishima, Kuniya Tanaka, Michael Bouvet, Itaru Endo, Fritz C. Eilber, Robert M. Hoffman

**Affiliations:** ^1^ AntiCancer, Inc., San Diego, CA, USA; ^2^ Department of Surgery, University of California, San Diego, CA, USA; ^3^ Department of Gastroenterological Surgery, Graduate School of Medicine, Yokohama City University, Yokohama, Japan; ^4^ Division of Hematology-Oncology, University of California, Los Angeles, CA, USA; ^5^ Department of Pathology, University of California, Los Angeles, CA, USA; ^6^ Division of Surgical Oncology, University of California, Los Angeles, CA, USA; ^7^ Department of Surgery, Yale University School of Medicine, New Haven, CT, USA; ^8^ Department of Pediatrics and Department of Orthopaedics, University of California, Los Angeles, CA, USA; ^9^ UCLA Sarcoma Program, Jonsson Comprehensive Cancer Center, University of California, Los Angeles, CA, USA; ^10^ PDOX Inc., San Diego, CA, USA

**Keywords:** palbociclib, linsitinib, patient-derived orthotopic xenograft, PDOX, Ewing's sarcoma

## Abstract

Ewing's sarcoma is a rare and aggressive malignancy. In the present study, tumor from a patient with a Ewing's sarcoma with cyclin-dependent kinase inhibitor 2A/B (*CDKN2A/B*) loss and *FUS-ERG* fusion was implanted in the right chest wall of nude mice to establish a patient-derived orthotopic xenograft (PDOX) model. The aim of the present study was to determine efficacy of cyclin-dependent kinase 4/6 (CDK4/6) and insulin-like growth factor-1 receptor (IGF-1R) inhibitors on the Ewing's sarcoma PDOX. The PDOX models were randomized into the following groups when tumor volume reached 50 mm^3^: G1, untreated control; G2, doxorubicin (DOX) (intraperitoneal (i.p.) injection, weekly, for 2 weeks); G3, CDK4/6 inhibitor (palbociclib, PD0332991, per oral (p.o.), daily, for 14 days); G4, IGF-1R inhibitor (linsitinib, OSI-906, p.o., daily, for 14 days). Tumor growth was significantly suppressed both in G3 (palbociclib) and in G4 (linsitinib) compared to G1 (untreated control) at all measured time points. In contrast, DOX did not inhibit tumor growth at any time point, which is consistent with the failure of DOX to control tumor growth in the patient. The results of the present study demonstrate the power of the PDOX model to identify effective targeted molecular therapy of a recalcitrant DOX-resistant Ewing's sarcoma with specific genetic alterations. The results of this study suggest the potential of PDOX models for individually-tailored, effective targeted therapy for recalcitrant cancer.

## INTRODUCTION

Sarcomas are a heterogeneous group of connective tissue malignancies of mesenchymal origin. They comprise approximately 1 percent of adult and 15 percent of pediatric malignancies. The most frequent site of primary sarcoma is the extremity, followed by the retroperitoneum and trunk. The most common site of metastasis is the lung. However, sarcoma can metastasize to almost any location or organ. There are over 50 known histological sub-types of sarcoma. Ewing's sarcoma is a rare malignancy in which *EWS-FLI1* is considered to be the causal translocation for 90% of cases [1]. Treatment for Ewing's sarcoma uses surgery, radiation, and chemotherapy but with poor outcome. Novel more effective treatment is necessary for this recalcitrant disease [2–7].

Palbociclib (PD0332991), a CDK4/6 inhibitor, has shown treatment efficacy for ovarian cancer, glioblastoma, and chordoma cell lines with *CDKN2A* loss [8–10]. Recently, palbociclib treatment efficacy for a patient with metastatic breast cancer with *CDKN2A* loss has been described. A clinical trial in patients with liposarcoma with *CDK4* amplification showed promising efficacy of palbociclib treatment [11].

Linsitinib (OSI-906) is a kinase inhibitor of both insulin receptor (IR) and insulin growth factor receptors (IGF-1R) [12]. Linsitinib was previously used to treat osteosarcoma cells and Ewing's sarcoma cells [13]. Linsitinib is being tested in a Phase III trial in adrenocortical carcinoma and in a Phase I/II clinical trial in ovarian cancer [14].

Clinically-relevant mouse models of sarcomas would permit evaluation of targeted molecular individualized therapy based on the genetic alternations of the patient's tumor. Our laboratory pioneered the patient-derived orthotopic xenograft (PDOX) nude mouse model with the technique of surgical orthotopic implantation (SOI). Our laboratory has developed PDOX models of all major tumor types including pancreatic [15–19], breast [20], ovarian [21], lung [22], cervical [23], colon [24–26] and stomach cancer [27] as well as mesothelioma [28] and sarcoma [6 29–31].

Recently, a patient tumor with high-grade undifferentiated pleomorphic soft-tissue sarcoma from a striated muscle was grown orthotopically in the right biceps femoris muscle of nude mice to establish a PDOX model. Tumor-targeting *S. typhimurium* A1-R followed by DOX eradicated the PDOX tumor in our laboratory [6].

A PDOX nude mouse model of follicular dendritic-cell sarcoma (FDCS) was also established in the biceps muscle of nude mice in our laboratory. The FDCS PDOX was resistant to both doxorubicin (DOX), as well as to NVP-BEZ235, dactolisib (BEZ), an experimental agent which is a dual pan-phosphoinositide 3-kinase-mammalian target of rapamycin inhibitor. However, in contrast to DOX and BEZ, the FDCS PDOX was sensitive to tumor-targeting *Salmonella typhimurium* A1-R [31].

In the present study, a Ewing's sarcoma patient with both *FUS-ERG* fusion [1, 32] and *CDKN2A/B* loss was studied. No patient with both these genetic alterations has been previously reported. Therefore, CDK4/6- and IGF-1R-inhibitors (Figure 1) were tested on this patient's tumor in the PDOX model (Figure 2).

**Figure 1:** Schematic representation of Palbociclib (PD0332991, CDK4/6 inhibitor) and Linsitinib (OSI-906, IGF-1R inhibitor) blockade CDK4/6 forms a complex with cyclin D which activates a cascade resulting in cell proliferation. Palbociclib inhibits CDK4/6 that is activated by the loss of *CDKN2A.* Linsitinib blocks IGF-1R which is activated by its ligands, IGF-1 or IGF-2, resulting in apoptosis blockade, and cell proliferation. IGF-1R: insulin-like growth factor-1 receptor; CDK: cyclin-dependent kinase.

**Figure 2:** Establishment of Ewing's sarcoma PDOX model **A.** After making a skin incision on the right chest wall of a nude mouse, the space between the pectoral muscle and intercostal muscle (arrow) was expanded. A 4 mm^3^ fragment of the patient tumor was implanted orthotopically into the space. **B.** The pectoral muscle and the skin were closed with a 6-0 nylon suture. Scale bar: 10 mm.

## RESULTS AND DISCUSSION

### Genetic alterations in the patient's tumor

Gene expression profiling (Foundation Medicine, Cambridge, MA) of the patient tumor revealed genetic alteration of *CDKN2A/B* loss and *FUS-ERG* fusion.

### Comparison of histology of original patient tumor and PDOX model

Histological analysis of the patient's tumor demonstrated an infiltrative proliferation of small round blue cells with round-to-avoid hyperchomatic nuclei, scanty eosinophilic-to-clear cytoplasm, and diffuse, membranous CD99 immunoreactivity. The PDOX tumor had a similar histomorphologic appearance similar to the original biopsy (Figure 3).

**Figure 3:** Histological comparison between patient original tumors and a PDOX tumor **A.** H & E staining of the resected patient original tumor and **B.** H & E staining of the untreated PDOX tumor. Scale bars: 50 μm.

### Palbociclib (PD0332991, CDK4/6 inhibitor) and Linsitinib (OSI-906, IGF-1R inhibitor) significantly inhibited tumor growth in the Ewing's sarcoma PDOX model

The PDOX models were randomized into the following groups when tumor volume reached 50 mm^3^: G1, untreated control; G2, DOX (intraperitoneal (i.p.) injection, weekly, for 2 weeks); G3, CDK4/6 inhibitor (palbociclib, PD0332991, per oral (p.o.), daily, for 14 days); G4, IGF-1R inhibitor (linsitinib, OSI-906, p.o., daily, for 14 days). DOX did not inhibit tumor growth, which is consistent with the failure of DOX to control tumor growth in the patient. Palbociclib significantly inhibited tumor growth compared to untreated control from day 8 to 22 (Figure 4, P > 0.01 at day-22). Linsitinib also significantly inhibited tumor growth compared to control from day 4 to 22 (Figure 4, P > 0.01 at day-22). On day 22, tumor volume was as follows: untreated control (G1) (209.8 ± 48.5 mm^3^); DOX (G2) (175.7 ± 79.9 mm^3^); palbociclib (G3) (74.3 ± 47.9 mm^3^); and linsitinib (G4) (101.0 ± 20.3 mm^3^).

**Figure 4:** Palbociclib (PD0332991, CDK4/6 inhibitor) and linsitinib (OSI-906, IGF-1R inhibitor) significantly inhibited tumor growth in a Ewing's sarcoma PDOX model Line graph shows tumor volume at each time point. Palbociclib significantly inhibited tumor growth compared to untreated control from day 8 to 22. Linsitinib also significantly inhibited tumor growth compared to control from day 4 to 22. In contrast, doxorubicin did not inhibit tumor growth at any time point. *P < 0.05, **P < 0.01 compared to untreated control. Error bars: ± 1 SD. *CDK:* cyclin-dependent kinase; IGF-1R: insulin-like growth factor-1 receptor; PDOX: patient-derived orthotopic xenograft.

Since *CDKN2A,* a tumor suppressor gene, suppresses CDK4/6 which stimulates cancer cells to cycle, loss of *CDKN2A* can result in increased cancer-cell proliferation. Incidence of *CDKN2A* loss in tumors of Ewing's sarcoma was reported to be relatively frequent with 11.2%. Palbociclib (PD0332991), a CDK4/6 inhibitor, had shown treatment efficacy for ovarian cancer, glioblastoma, and chordoma cell lines with *CDKN2A* loss [8–10]. Recently, palbociclib treatment efficacy for a patient with metastatic breast cancer with *CDKN2A* loss has been described [34]. A clinical trial in patients with liposarcoma with *CDK4* amplification showed promising efficacy of palbociclib treatment [11]. Palbociclib treatment efficacy in the present study is likely through suppression of the CDK4/6 pathway which was activated by *CDKN2A* loss (Figure 1).

The findings of *CDKN2A/B* loss offered a clue that this tumor may be succeptible to CDK4/6 inhibition, which is normally inhibited by *CDKN2A/B* and suggests that the cell cycle is a viable target in Ewing's sarcoma [34, 35].

The patient's tumor was characterized by a *FUS-ERG* fusion gene as well as the *CDKN2A/B* loss. Ewing's sarcoma is a rare small round blue-cell tumor that is mostly characterized by translocations involving *EWSR1* and members of the ETS transcription factor family. In recent years, Ewing's sarcoma like small round blue cell tumors have been characterized by non-canonical translocations including *CIC-DUX4* [36] and *FUS-ERG* [32, 37]. It is felt that these non-canoncial Ewing's sarcomas make up a portion of the group of atypical Ewing's sarcomas. Because of the rarity of *FUS-ERG* in Ewing's sarcomas, the prognosis, treatment and molecular biology of this genetic alteration is poorly understood. The development of PDOX models will help to better study and define this disease.

Currently there are no therapies that have been developed that reliably inhibit ERG fusion proteins. This rare *FUS-ERG* transgene has also been noted in ALL and AML and found to modulate the retinoic acid pathway in AML [38]. In addition, Cironi et. al. [39] demonstrated that this fusion gene upregulated IGF-1 in AML indicating that this may be a candidate target for diseases with the *FUS-ERG* transgenes. Other studies in leukemia point to a possible role for PIM1 and MAPK inhibitors for malignancies with *ERG* transgenes [40]. The IGF-1R pathway promotes proliferation and prevents apoptosis of cancer cells through activation of phosphatidylinositol 3-kinase (PI3K) and mitogen-activated protein kinase (MAPK) pathways [41]. Consistent expression of IGF-1R was observed both in Ewing's sarcoma cell lines and patient tissue [42, 43]. In a Phase II study for patients with Ewing's sarcoma, measurable treatment response to an IGF-1R inhibitor was demonstrated [42]. In the present study, the IGF-R inhibitor linsitinib essentially arrested the Ewing's sarcoma (Figure 4), suggesting further study and use of this inhibitor in sarcoma.

## CONCLUSIONS

We report here significant efficacy of CDK4/6 and IGF-1R inhibitors on a rare Ewing's sarcoma with *FUS-ERG* fusion and *CDKN2A/B* loss in a PDOX model. The results can be used to tailor further treatment for this patient.

Until 2003, all of the reported Ewing tumors involved rearrangement of the *EWS* gene, at 22q12, with an *ETS*-family transcription factor. In 2003, four Ewing's tumor cases were reported that had joined chromosome bands 16p11 and 21q22. Detailed genetic analysis of two of the cases demonstrated how this rearrangement resulted in the fusion of the *FUS* gene at 16p11 to the *ERG* gene at 21q22 [32].

The fusion proteins could possibly comprise the transactivation domain of *FUS* and the DNA-binding domain of transcription factor *ERG*; thus *FUS/ERG* may be an aberrant transcription factor [32].

The four Ewing's tumor cases previously described and the present case may represent a novel type of Ewing's tumor in which 22q12 is not rearranged, and the primary translocation involves chromosomes 16 and 21 [32].

Cironi et al [39] observed in transfection studies that *FUS/ERG* activated the IGF-1 promoter and induced IGF-1 expression. This is consistent with the results of the present study that targeting the IGF-IR inhibited the Ewing sarcoma PDOX with the *FUS/ERG* fusion.

Palbociclib, a small-molecule inhibitor of cyclin-dependent kinases 4 and 6 [8–10], was recently approved by the FDA for HER2-negative breast cancer. *CDKN2A* (p16) is a negative regulator of CDK 4 and 6. Previously a patient with metastatic estrogen receptor- positive, HER2-negative breast cancer with *CDKN2A* loss responded to palbociclib, as briefly described above, which is consistent with the results of the present study, where palbociclib inhibited the Ewing's sarcoma PDOX, which lost *CDKN2A*, by targeting CDK4/6 [33].

In a previous study from our laboratory, fluorophore-conjugated IGF-1R antibodies selectively visualized metastatic colon cancer [44]. Future studies will use the IGF-IR antibodies to detect metastasis in PDOX models of Ewing's sarcoma to enable determination of efficacy of molecular inhibitors on metastasis as well as the primary tumor.

Previously developed concepts and strategies of highly selective tumor targeting can take advantage of molecular targeting of tumors, including tissue-selective therapy which focuses on unique differences between normal and tumor tissues [45–50].

## MATERIALS AND METHODS

### Mice

Athymic *nu/nu* female nude mice (AntiCancer Inc., San Diego, CA), 4–6 weeks old, were used in this study. All animal studies were conducted with an AntiCancer Institutional Animal Care and Use Committee (IACUC)-protocol specifically approved for this study and in accordance with the principals and procedures outlined in the National Institutes of Health Guide for the Care and Use of Animals under Assurance Number A3873-1. In order to minimize any suffering of the animals the use of anesthesia and analgesics were used for all surgical experiments. Animals were anesthetized by subcutaneous injection of a 0.02 ml solution of 20 mg/kg ketamine, 15.2 mg/kg xylazine, and 0.48 mg/kg acepromazine maleate. The response of animals during surgery was monitored to ensure adequate depth of anesthesia. The animals were observed on a daily basis and humanely sacrificed by CO_2_ inhalation when they met the following humane endpoint criteria: severe tumor burden (more than 20 mm in diameter), prostration, significant body weight loss, difficulty breathing, rotational motion and body temperature drop. Animals were housed in a barrier facility on a high efficiency particulate arrestance (HEPA)-filtered rack under standard conditions of 12-hour light/dark cycles. The animals were fed an autoclaved laboratory rodent diet.

### Patient-derived tumor

The Ewing's sarcoma tumor from the right chest wall of a female patient was resected by JY in the Department of Surgery, University of California, Los Angeles (UCLA). Written informed consent was provided by the patient, and the Institutional Review Board (IRB) of UCLA approved this experiment. Neoadjuvant chemotherapy with DOX, vincristine, and cyclophosphamide, was previously administered to the patient.

### Establishment of PDOX model of soft-tissue Ewing's sarcoma

A fresh tumor tissue sample from the Ewing's sarcoma from the right chest wall was obtained and transported immediately to the laboratory of AntiCancer on ice. The sample was minced into 5 mm fragments. The tumor fragments were implanted subcutaneously in nude mice. Seven weeks later, the implanted tumors grew to approximately 10 mm in diameter. The established tumors were harvested and minced into 4 mm^3^ fragments. Mice were anethesized with the ketamine mixture. A 10 mm skin incision was made on the right chest wall. The PDOX model was established by implanting a single tumor fragment orthotopically into the layer between the pectoral muscle and intercostal muscle in the right chest wall of the nude mouse. The wound was closed with a 6-0 nylon suture (Ethilon, Ethicon, Inc., NJ) (Figure 2).

### Treatment study design in the PDOX model of sarcoma

*Experimental protocol*: G1: untreated control (n = 6); G2: treated with doxorubicin (i.p., 3 mg/kg, weekly, 2 weeks, n = 6); G3: treated with palbociclib (p.o., 100 mg/kg, daily, 14 days, n = 6); G4: treated with linsitinib (p.o., 25 mg/kg, daily, 14 days, n = 6). When tumor volume reached 50 mm^3^, treatment started. Tumor length and width were measured twice in a week. Tumor volume was calculated with the following formula: Tumor volume (mm^3^) = length (mm) × width (mm) × width (mm) × 1/2. Data are presented as mean ± SD. Tumor growth inhibition was defined as following equation reported by Stebbing et al. [51]: Tumor growth inhibition (%) = (1 − (T_22_ − T_1_) / (C_22_ − C_1_)) × 100. T_1_, average treated tumor volume on day 1; T_22_, average treated tumor volume on day 22; C_1_, average control tumor volume on day 1; C_22_, average control tumor volume on day 22. All treated mice were followed up until day 22.

### Histological examination

Fresh tumor samples were fixed in 10% formalin and embedded in paraffin before sectioning and staining. Tissue sections (5 μm) were deparaffinized in xylene and rehydrated in an ethanol series. Hematoxylin and eosin (H&E) staining was performed according to standard protocol. Histological examination was performed with a BHS system microscope (Olympus Corp., Tokyo, Japan). Images were acquired with INFINITY ANALYZE software (Lumenera Corporation, Ottawa, Canada) [6, 31].

### Statistical analysis

SPSS statistics version 21.0 was used for all statistical analyses (IBM, New York City, NY, USA). Significant differences for continuous variables were determined using the Mann-Whitney U test. Line graphs expressed average and error bar showed SD. A probability value of *P* ≤0.05 was considered statistically significant.
